# Study on Factors Associated with High Myopia CNV in Aqueous Humor and Serum

**DOI:** 10.1155/2022/8592729

**Published:** 2022-04-30

**Authors:** Yi Fan Xia, Jing Wei

**Affiliations:** Henan University of Science and Technology, Luoyang, Henan Province 471000, China

## Abstract

**Objective:**

The objective is to investigate the relationship and correlation between PEDF and TGF-*β* in aqueous humor and serum and high myopia CNV lesions.

**Methods:**

For each group of patients (namely, group A: patients with high myopia CNV (mCNV); group B: patients with high myopia without CNV; group C: patients with CNV caused by other eye diseases; and group D (control group): patients with simple cataract (without CNV and high myopia)), 20 patients were collected. A total of 40 patients have been collected since the beginning of the study in December 2020, including 7 patients in group A, 13 patients in group B, 10 patients in group C, and 10 patients in group D. Serum and aqueous humor samples were collected, and PEDF and TGF-*β* levels in serum and aqueous humor were detected by enzyme-linked immunosorbent assay (ELISA). SPSS 26.0 statistical software was used to process the data. Independent sample *t*-test was used to compare the data of the same factor in the same group between serum and aqueous humor. Comparisons of the same factors between different groups were performed using a one-way analysis of variance (ANOVA). Correlation analysis was conducted by the Pearson correlation coefficient test. *P* < 0.05 indicated that the difference was statistically significant.

**Results:**

There were no significant differences in age, gender, and course of disease among all groups (*P* > 0.05). The concentration of PEDF in aqueous humor in group A and group C was higher than that in group B and group D. There was no significant correlation between serum PEDF content and the above-mentioned diseases. The concentration of TGF-*β* in aqueous humor in groups A, B, and C was significantly higher than that in group D. However, there was no significant correlation between TGF-*β* content in serum and the above-mentioned diseases. There was no significant correlation between aqueous humor and serum PEDF. There was no significant correlation between the content of TGF-*β* in aqueous humor and serum.

**Conclusion:**

TGF-*β* in aqueous humor may be involved in the development of high myopia and intraocular CNV disease. However, PEDF in aqueous humor may be involved in the development of intraocular CNV disease and has no significant correlation with high myopia. At the same time, TGF-*β* and PEDF in serum had no significant correlation with high myopia and intraocular CNV disease. There was no significant correlation between the concentrations of TGF-*β* and PEDF in aqueous humor and serum.

## 1. Introduction

High myopia accounts for 153 million of the world's population [1], making it a serious public health problem in the world. The prevalence of high myopia varies greatly among different countries, among which the incidence is higher in Southeast Asian countries. The survey shows that high myopia, especially very high myopia, has increased significantly over the past 15 years, with Seoul having the highest prevalence of high myopia (21.61% in 2012), followed by Shanghai (19.5 percent in 2012), Zhejiang (15.4 percent in 2014), Shandong (14 percent in 2013), Beijing (6.69 percent in 2015), and Jeju (6.8 percent in 2013). Taiwan, China, had a staggering 38 percent prevalence of high myopia, a recent systematic review predicted. By 2050, there are an estimated 4.758 billion people with myopia (49.8% of the world's population) and 938 million people with high myopia (9.8% of the world's population) [2]. High myopia is a serious but often underestimated eye condition. As a disease that crosses genders, ages, and races, it is characterized by low awareness and high incidence, and many problems are still in the research stage.

The incidence and prevalence of myopic choroid neovascularization (mCNV) vary greatly. The occurrence probability of CNV in patients with high myopia is 9 times higher than that in normal people. The prevalence rate of CNV is 5.2%-11.3% in patients with high myopia. Bleeding and edema between retinal tissues caused by CNV are common complications leading to visual function loss in patients with high myopia, which greatly reduces the vision-related quality of life of patients. Degenerative CNV is often accompanied by retinal scar fibrosis, atrophy, and thinning of pigment epithelial Bruch membrane complex, leading to irreversible low vision [3]. Therefore, it is very important to study its risk factors for the prevention and treatment of this disease. At present, high myopia CNV is recognized as a disease because of the following: (1) the formation of CNV is a compensatory mechanism due to choroid thinning and insufficient blood supply, and (2) in patients with abnormal axial extension, it leads to the pole of the structure, the choroid and retinal thickness and corresponding RPE layer, the thickness of the photoreceptor cell layer, and with the axial extension and thinning, causing the appearance of the paint crack, lacquer cracks for CNV, and inflammation factors, such as fiber cells by choroid retinal internal growth to provide a space [6]. With the development of the disease course, CNV may evolve into fibrovascular scar tissue under the regulation of cytokines and the body's repair and gradually develop into atrophy foci with further degeneration. Without treatment, the vision of most patients with myopic CNV will further deteriorate and may lead to blindness. A large number of studies have shown that the generation and development of CNV in high myopia is related to the changes of many cytokines [7, 8].

Previous studies have shown that a variety of growth factors, proteolytic enzymes, and cell adhesion molecules are involved in the process of neovascularization as follows [9, 10]:

1. The balance between stimulators and inhibitors maintaining normal vascular metabolism is broken; the activity of angiogenic factors (TGF-*β*) is upregulated so that inner skin cells and pericytes are activated and cell division and proliferation are accelerated
2. The levels of metalloproteinase, plasminogen activator, serine protein hydrolase, and other hydrolases in vascular basement membrane were upregulated to degrade the basement membrane and extracellular matrix
3. The expression of adhesion molecules on the endothelial cell membrane is upregulated. For example, integrin 3 induces endothelial cells to invade the stromal layer of surrounding tissues and proliferate and migrate by stimulating calcium signal regulation pathway
4. The expression of various receptor molecules promoting vascular endothelial growth factors, such as TGF-*β* receptor Flt-1 and angiopoietin receptor Tie-1 and Tie-2, also increased accordingly. These receptors combined with growth factors to promote the assembly of endothelial cells to form lumen, tube climbing, and vascular network
5. Under the action of angiopoietin-1 and angiopoietin-2, vascular remodeling is completed by promoting or relaxing the interaction between endothelial cells and their surrounding supporting cells. It can be seen that “the balance between stimulators and inhibitors maintaining normal vascular metabolism is broken” is an important link in neovascularization.

During the formation of CNV, TGF-*β* and bFGF are the main angiogenic factors and play an induction and stimulation role in the formation of CNV [10, 11]. However, TGF-*β* and other inhibitory factors that inhibit endothelial cell proliferation are also expressed in experimental CNV formation [12]. These results suggest that CNV formation is also regulated by two reactive cytokine systems, angiogenic stimulator and inhibitory factor, and the imbalance between them is the main cause of CNV formation. Therefore, it has become one of the focuses of basic and clinical research on CNV to study the expression of related cytokines in the pathogenesis of CNV and their roles in the formation of CNV and to regulate their expression levels according to the biological activities and physiological functions of various key factors, to intervene in neovascularization. Therefore, in this study, the contents of PEDF and TGF-*β* in aqueous fluid and serum of CNV patients with high myopia were detected at the clinical level, and clinical data were collected to evaluate the relationship between the content and disease activity. This study will reveal the relationship between PEDF and TGF-*β* and the development of high myopia CNV as well as the correlation PEDF between and TGF-*β*, hoping to perfect new drug targets for the diagnosis and treatment of high myopia CNV.

## 2. Methods

### 2.1. Participant

For each group of patients (namely, group A: patients with high myopia CNV (mCNV); group B: patients with high myopia without CNV; group C: patients with CNV caused by other eye diseases; and group D (control group): patients with simple cataract (without CNV and high myopia)), 20 patients were collected. A total of 40 patients have been collected in December 2020 to October 2021, including 7 patients in group A, 13 patients in group B, 10 patients in group C, and 10 patients in group D. The male to female ratio was 22 : 18, and the mean age was 64.1 ± 7.2 years in Figure 1.

### 2.2. Inclusion Criteria

The inclusion criteria as follows: (1) according to the diagnosis of high myopia, with equivalent spherical lens ≥ -6.00d or axial length ≥26 mm, for those with lens surgery or corneal surgery, preoperative refractive data were used. The medical records of each patient's first visit were used for analysis. (2) All patients had high myopia in both eyes. (3) The fundus showed high myopia: Leopard-shaped fundus, lacquer crack, periodical choroidal atrophy, and posterior scleral staphyloma. (4) It is consistent with the CNV diagnosis of high myopia: fundus angiography and OCT examination suggest the existence of choroidal neovascularization in the macular area. (5) CNV was found in one or both eyes.

### 2.3. Exclusion Criteria

The exclusion criteria are as follows: (1) complicated with corneal disease, obvious cataract opacity, vitreous volume blood, and other refractive media opacity; (2) there were amblyopia, glaucoma, retinal detachment, retinal vein occlusion, fundus hemorrhage, diabetic retinopathy, and systemic diseases; (3) any one of the eyes of the patient has undergone internal eye surgery such as retina; (4) retinal choroidal neovascularization caused by other clear reasons (such as trauma, infection, age, idiopathic polypoid choroidal angiopathy, and choroidal hemangioma) shall be excluded; and (5) monocular high myopia.

### 2.4. Serum Sample Collection

On the day of admission, 3~4 ml of elbow vein blood was drawn in the morning under the resting fasting state, mixed in the test tube containing coagulant + separating gel, and separated by low-temperature ultracentrifuge (4°C, 2000 r/min centrifugation, 10 min); 0.3~0.4 ml of serum was taken and put into 0.5-ml sterile Eppendorf tube, labeled, and stored in the -80°C low-temperature refrigerator for examination.

### 2.5. Aqueous Humor Sample Collection

During ophthalmic surgery, all patients entered the anterior chamber from the corneal limbal puncture port with a 1-ml syringe with No. 25 needle, slowly extracted 0.15~0.2 ml of undiluted aqueous humor, avoided contact with the retina, lens, and corneal endothelium, immediately injected into 0.5-ml sterile Eppendorf tube, and marked and stored in -80°C ultra-low-temperature refrigerator for examination.

### 2.6. Elisa Assay

The contents of PEDF and TNF*β* in serum and aqueous humor of each group were detected by enzyme-linked immunosorbent assay (ELISA). Centrifuge each tube for three minutes when using the kit for the first time. The specimen was removed from the refrigerator and placed at room temperature for 10 min for testing. All operations were carried out in strict accordance with the kit instructions.

### 2.7. Statistical Analysis

SPSS26.0 statistical software was used for correlation analysis of the data. The statistical data were normally distributed, and the measurement data were expressed as mean ± standard deviation (*X* ± *S*). The mean values of the four groups were tested for homogeneity of variance, and one-way ANOVA was used. ANOVA was used to analyze the relationship between TGF-*β* and PEDF in aqueous humor and serum and four groups of data. Pearson correlation analysis was conducted for the cytokine levels between aqueous humor and serum in each group, and *P* < 0.05 was considered statistically significant.

## 3. Results

### 3.1. General Information

There were no significant differences in age, gender, and course of disease among all groups (*P* > 0.05) in Table 1.

### 3.2. Levels of PEDF in Aqueous Humor and Serum

The concentration of PEDF in aqueous humor in group A and group C was higher than that in group B and group D, indicating that PEDF may be involved in the development of the CNV process, but there was no significant correlation with high myopia. There was no significant correlation between serum PEDF content and the above-mentioned diseases, indicating that serum PEDF had no significant effect on intraocular diseases in Table 2.

### 3.3. TGF-*β* Levels in Aqueous Humor and Serum

The concentration of TGF-*β* in aqueous humor in groups A, B, and C was significantly higher than that in group D, suggesting that TGF-*β* may be involved in the development of high myopia and intraocular CNV. However, there was no significant correlation between TGF-*β* content in serum and the above-mentioned diseases, indicating that TGF-*β* in serum had no significant effect on intraocular diseases in Table 3.

### 3.4. Correlation Analysis of PEDF Concentration between Aqueous Humor and Serum in each Group

There was no significant correlation between aqueous humor and serum PEDF, indicating that the content of PEDF in aqueous humor was not affected by the serum in Table 4.

### 3.5. Correlation Analysis of TGF-*β* Concentration between Aqueous Humor and Serum in each Group

There was no significant correlation between the content of TGF-*β* in aqueous humor and serum, indicating that the content of TGF-*β* in aqueous humor was not affected by the serum in Table 5.

## 4. Discussion

High myopia (HM) is one of the most serious common diseases of all refractive errors, and the occurrence of choroidal neovascularization (CNV) in the macular region is an important cause of vision loss in HM patients. Because of its relatively irreversible damage to visual function, it often causes great trouble to patients' life and works. The cause of high myopia with CNV is unclear. Many theories have been used to explain the causes of CNV, but all of them have shortcomings. There are mainly the following kinds [2]: (1) The choroid thickness of myopia patients with ocular axis lengthening and abnormal posterior pole structure becomes thinner, and at the same time, the thickness of the RPE layer and the corresponding photoreceptor cell layer may also decrease in the same proportion. Choroid becomes thinner over time with secondary outer retinal ischemia. Due to the tearing and rupture of the pigment epithelium Bruch membrane choroidal capillary wall under mechanical action and the function of tissue self repair, paint like cracks are formed, creating a certain space, providing tissue space for neovascularization, pericytes, fibroblasts, and inflammatory cells to enter the retina from the choroid, and providing conditions for the occurrence of CNV [3]. The paint crack (2) most high myopia, but only a handful of progress for the CNV, so there may be other factors involved in the formation of myopia CNV [13]. For example, due to high myopia, the choroid in the macular area is significantly thinner than that in normal people, the thinning choroidal capillaries are reduced or even completely lost, so the perfusion is reduced, resulting in choroidal ischemia and hypoxia. Severe choroid atrophy leads to decompensation of the retinal pigment epithelium, gradual thinning and atrophy of the retinal pigment epithelium, and disturbance or defect of photoreceptors, and retinal outer layer leads to upregulation of vascular endothelial growth factor, leading to choroid neovascularization [14]. (3) Studies have shown that high myopia CNV is associated with some inflammatory markers. Studies have found that the occurrence of myopia CNV is related to the increase of inflammatory factors, indicating that inflammatory factors play a certain role in the occurrence and development of CNV [15]. The pathological course of HIGH myopia CNV is generally divided into three courses. At first, choroidal neovascular directly destroys photoreceptor cells through their physical injury and bleeding, cytokines, and inflammatory factors brought by incomplete blood vessels, leading to the loss of central visual function [16]. With the development of the disease course, CNV gradually moved to the fibrous scar stage, called Fuchs spot, due to its repair function and the influence of various inflammatory factors. Eventually, choroidal neovascularization gradually degenerates, and atrophy foci are formed, which is the key to permanent vision loss [17]. Therefore, early detection and early treatment of myopia CNV are important.

PEDF was originally isolated from the culture medium of retinal pigment epithelial RPE [18]. Its molecular weight is 50 kD, located on chromosome 17p13 [19]. PEDF can be produced in multiple parts of the eye: RPE cells can secrete PEDF into the Inter photoreceptor matrix (IPM), which has a physiological role in protecting the retina. PEDF can be produced by the pigment-free layer of ciliary epithelium, corneal epithelial cells, and ganglion cells [20]. PEDF is also found in vitreous and aqueous humor, as well as in the human brain, cerebrospinal fluid, plasma, liver, testis, ovary, placenta, and other tissues. PEDF can inhibit a variety of angiogenesis inducers, including platelet-derived factors, vascular endothelial growth factor, interleukin-8, and acid fibroblast growth factor. PEDF is one of the most effective angiogenesis inhibitors.

PEDF can induce apoptosis of activated vascular endothelial cells and inhibit neovascularization. It has been reported that PEDF may induce apoptosis of activated vascular endothelial cells so that vascular endothelial cells cannot respond to hypoxia-induced neovascularization signals [21]. The results of this study showed that the concentration of PEDF in aqueous humor in group A and group C was higher than that in group B and group D, indicating that PEDF may be involved in the development of the CNV process, but there was no significant correlation with high myopia. There was no significant correlation between serum PEDF content and the above-mentioned diseases, indicating that serum PEDF had no significant effect on intraocular diseases.

TGF-*β* is a kind of multiskin regulatory protein with a variety of biological activities, involved in regulating cell proliferation, differentiation, extracellular matrix (ECM) deposition, degradation, and other physiological and pathological processes. TGF-*β* plays an important regulatory role in tissue development, angiogenesis, and injury repair [23]. TGF-*β* can promote the apoptosis of vascular endothelial cells [24] and is a highly active inhibitory factor of endothelial cell proliferation [24–26]. Mammalian TGF-*β* has three isomers with 70%-80% homology in nucleotide sequence [22, 27] and similar biological functions. Among them, TGF-*β* accounts for the highest proportion (>90%) in somatic cell lines and has the strongest activity [28]; its inhibitory effect on endothelial cells is greater than TGF-*β*, and it is the main cytokine promoting ECM formation, so it has become the focus of our study. In this study, the concentration of TGF-*β* in aqueous humor in groups A, B, and C was significantly higher than that in group D, suggesting that TGF-*β* may be involved in the development of high myopia and intraocular CNV. However, there was no significant correlation between TGF-*β* content in serum and the above-mentioned diseases, indicating that TGF-*β* in serum had no significant effect on intraocular diseases.

It is known that a variety of angiogenesis inhibitors are expressed in the process of neovascularization, such as angiostatin, endostatin, thrombospondin, and platelet factor 4. PEDF is currently recognized as the most active angiogenesis inhibitor, while TGF-*β* is an important regulator of cell proliferation and differentiation, extracellular matrix deposition, and degradation. Both PEDF and TGF-*β* had a strong inhibitory effect on endothelial cells. In this study, linear correlation analysis showed a negative correlation between PEDF and TGF-*Β* levels in the aqueous humor of A patients. Therefore, we speculated that the decrease of PEDF level and the increase of TGF-*β* level in the aqueous humor may promote the generation of retina neovascularization.

All the experimental methods used in the study are widely used in domestic and foreign research methods; the technology is very mature. The central laboratory of the First Affiliated Hospital of Henan University of Science and Technology, the New District Medical Experiment Center, and the School of Medicine of Henan University of Science and Technology have the experimental conditions and instruments needed to carry out this research. However, there are few studies on the relationship between the contents of TGF-*β* and PEDF in aqueous humor and CNV in high myopia at home and abroad, and the relationship between the contents of TGF-*β* and PEDF in aqueous humor and serum is not clear, as well as whether the contents of TGF-*β* and PEDF in serum and aqueous humor are related is controversial. We will continue to improve it in the follow-up study.

## 5. Conclusion

The imbalance of the expression of vascular inhibitory and stimulatory factors in patients of HM-CNV is an important factor affecting the occurrence and development of the disease. If the imbalance of the expression of factors in A patients can be detected early, it may play a positive role in the prevention of HM-CNV. If the abnormal expression of factors related to intraocular factors can be found in the blood of HM-CNV patients at an early stage, we can intervene in the disease at an early stage and prevent its further development, which will be of great help to the early diagnosis and treatment of the disease. In this study, TGF-*β* in aqueous humor may be involved in the development of high myopia and intraocular CNV disease. However, PEDF in aqueous humor may be involved in the development of intraocular CNV disease and has no significant correlation with high myopia. At the same time, TGF-*β* and PEDF in serum had no significant correlation with high myopia and intraocular CNV disease. There was no significant correlation between the concentrations of TGF-*β* and PEDF in aqueous humor and serum. Therefore, the study of related factors in serum and aqueous humor of HM-CNV patients is the main direction of our future work..

## Figures and Tables

**Figure 1:** Research flow chart.

**Table 1:** General information.

Group	*n*	Sex		Age	Course of disease
		Male	Female		
Group A	7	4	3	62.3 ± 8.4	3.7 ± 1.2
Group B	13	7	6	63.5 ± 5.9	41.3 ± 3.7
Group C	10	5	5	64.9 ± 7.6	2.6 ± 4.8
Group D	10	6	4	52.5 ± 6.6	—

**Table 2:** PEDF levels in serum and aqueous humor (*x* ± *s*).

Group	*n*	PEDF (pg/ml)	
		Aqueous humor	Serum
Group A	7	458.0 ± 8.6	462.8 ± 10.1
Group B	13	416.0 ± 7.8	470.0 ± 9.0
Group C	10	496.0 ± 9.8	471.7 ± 10.5
Group D	10	412.0 ± 9.9	468.4 ± 13.0

**Table 3:** TNF-*β* levels in serum and aqueous humor (*x* ± *s*).

Group	*n*	TGF-*β* (pg/ml)	
		Aqueous humor	Serum
Group A	7	522.7 ± 24	472.8 ± 10.1
Group B	13	476.5 ± 9.3	479.0 ± 9.0
Group C	10	480.2 ± 13.4	476.7 ± 10.5
Group D	10	403.4 ± 28.1	477.4 ± 13.0

**Table 4:** Correlation analysis of PEDF concentration between aqueous humor and serum in each group.

	PEDF	Group
PEDF in aqueous humor		
Pearson	1	-.625∗∗
Sig.		-.818
*n*	40	40
PEDF in serum		
Pearson	-.625∗∗	1
Sig.	-.818	
*n*	40	40

**Table 5:** Correlation analysis of TGF-*β* concentration between aqueous humor and serum in each group.

	TGF*-β*	Group
TGF-*β* in aqueous humor		
Pearson	1	-.828∗∗
Sig.		-.325
*n*	40	40
TGF-*β* in serum		
Pearson	-.828∗∗	1
Sig.	-.325	
*n*	40	40

## Data Availability

No data were used to support this study.
